The article "Study on the Mechanism of Huanglian Jiedu Decoction in Treating Dyslipidemia Based on Network Pharmacology" was published in 2022. Journal: J Healthc Eng.

# Study on the Mechanism of Huanglian Jiedu Decoction in Treating Dyslipidemia Based on Network Pharmacology

**DOI:** 10.1155/2022/2457706

**Published:** 2022-08-24

**Authors:** Zhaohui Gong, Rong Li, Shulin Chen, Hui Wu, Yinhe Cai, Junlong Li, Xinjun Zhao, Qingmin Chu, Chuanjin Luo, Lijin Qing, Nan Li, Wei Wu

**Affiliations:** ^1^Department of Cardiovascular, The First Affiliated Hospital, Guangzhou University of Chinese Medicine, Guangzhou 510405, China; ^2^The First Clinical Medical College, Guangzhou University of Chinese Medicine, Guangzhou 510405, China; ^3^Department of Rheumatology, the First Affiliated Hospital of Guangzhou University of Chinese Medicine, Guangzhou 510405, China; ^4^Formula-Pattern Research Center, School of Traditional Chinese Medicine, Jinan University, Guangzhou 510632, China

## Abstract

**Objective:**

This study aimed to determine the active ingredients of Huanglian Jiedu decoction (HLJDD) and the targets for treating dyslipidemia through network pharmacology to facilitate further application of HJJDD in the treatment of dyslipidemia.

**Methods:**

Potential drug targets for dyslipidemia were identified with a protein-protein interaction network. Gene ontology (GO) enrichment analysis and KEGG pathway analysis were performed to elucidate the biological function and major pathways involved in the HLJDD-mediated treatment of dyslipidemia.

**Results:**

This approach revealed 22 components, 234 targets of HLJDD, and 221 targets of dyslipidemia. There were 14 components and 31 common targets between HLJDD and dyslipidemia treatment. GO enrichment analysis showed that these targets were mainly associated with the response to DNA-binding transcription factor activity, lipid localization and storage, reactive oxygen species metabolic process, and inflammatory response. The results of KEGG analysis indicated that the AGE-RAGE, NF-*κ*B, HIF-1, IL-17, TNF, FoxO, and PPAR signalling pathways were enriched in the antidyslipidemic action of HLJDD.

**Conclusion:**

This study expounded the pharmacological actions and molecular mechanisms of HLJDD in treating dyslipidemia from a holistic perspective, which may provide a scientific basis for the clinical application of HLJDD.

## 1. Introduction

Dyslipidemia is a major risk factor for atherosclerotic cardiovascular disease (CVD), which accounts for more than half of all noncommunicable diseases and has become the leading cause of death worldwide [1]. It has been reported that about one-third of adults in the United States had dyslipidemia [2]. Studies in 2014–2019 revealed a consistently high prevalence of dyslipidemia in China, ranging from 33.8 to 43% among adults of middle or senior ages [3]. Moreover, recent studies have shown that the incidence of dyslipidemia among children and adolescents is also increasing annually [4].

The article "Study on the Mechanism of Huanglian Jiedu Decoction in Treating Dyslipidemia Based on Network Pharmacology" was published in 2022. Journal: J Healthc Eng.

The therapeutic strategy for patients with dyslipidemia depends on their coronary artery disease risk. For patients at high risk, drug therapy combined with specific healthy lifestyle changes should be administered immediately. For those at moderate or low risk, specific healthy lifestyle changes should be promoted, and if the lipid levels are not targeted, drug therapy should be added. The choice of dyslipidemia-regulating medications depends on the major lipid abnormality and includes statins, resins, fibrates, and niacin [5].

As an important aspect of the complementary and alternative medical system, traditional Chinese medicine (TCM) has been widely used in treating dyslipidemia for centuries. In TCM, dyslipidemia can be classified as “phlegm,” “wet,” or “blood turbidity,” which is caused by overeating greasy food, dysfunction of transportation, transformation of the spleen and stomach, stagnation of qi, and phlegm dampness [6]. Many herbs such as Rhizoma Coptidis (Huanglian), Radix Scutellariae (Huangqin), *Rheum officinale* (Dahuang), red yeast rice (Hongqu), and Fructus Crataegi (Shanzha) are frequently used in the treatment of hyperlipidemia and achieve significant effects in regulating blood lipids [7]. Many herbal formulas such as Da Chaihu decoction [8], Erchen decoction [9], Gegen Qinlian decoction [10], and Wendan decoction [11] also regulate dyslipidemia. These data suggest that TCM medications have a good effect on treating dyslipidemia.

Huanglian Jiedu decoction (HLJDD) is an herbal formula that originates from Zhou Hou Bei Ji Fang and was developed by Ge Hong and consists of 4 herbs: Fructus Gardeniae (FG, Zhizi), Radix Scutellariae (RS, Huangqin), Rhizoma Coptidis (RC, Huanglian), and Cortex Phellodendri (CP, Huangbai). Based on the TCM theory, multiple herbs in one formula should operate cooperatively. It has been reported that one of the aetiologies of dyslipidemia is heat toxicity, and HLJDD is able to clear heat and remove toxicity. Several basic studies have also shown that HLJDD has a certain effect on dyslipidemia [12, 13]. Therefore, HLJDD, alone or combined with other drugs (herbal formulas or Western medicine), has the potential to be a drug for dyslipidemia. However, its pharmacological mechanism has not been clarified completely. Therefore, the network pharmacology method was used to explore the impact of HLJDD on dyslipidemia and its pharmacological mechanism from another point of view.

## 2. Methods

The study strategy is illustrated in Figure 1.

### 2.1. Screening for the Targets of HLJDD Ingredients

The components of HLJDD, namely, Fructus Gardeniae, Radix Scutellariae, Rhizoma Coptidis, and Cortex Phellodendri, were searched in the TCMSP database (https://tcmspw.com/tcmsp.php, 2021/06/01), with oral bioavailability (OB) ≥ 30%, drug likeness (DL) ≥ 0.18, and drug half-life (HL) ≥ 4 h used as screening criteria to screen for targets of corresponding ingredients. Then, the UniProt database (https://www.uniprot.org/, 2021/06/01) was used for target correction, with species restricted to “*Homo sapiens*,” and the target proteins were transformed into corresponding genes.

The article "Study on the Mechanism of Huanglian Jiedu Decoction in Treating Dyslipidemia Based on Network Pharmacology" was published in 2022. Journal: J Healthc Eng.

### 2.2. Screening for the Targets of Dyslipidemia

The targets of dyslipidemia treatment were collected from the GeneCards (https://www.genecards.org/, 2021/06/16), OMIM (https://omim.org/, 2021/06/16), PharmGKB (https://www.pharmgkb.org/, 2021/07/20) (http://db.idrblab.net/ttd/, 2021/07/20), and DrugBank (https://go.drugbank.com/, 2021/08/22) databases, as well as the therapeutic target database (TTD).

### 2.3. Construction of the Herb-Component-Target Network

Herbs, components, and targets of HLJDD were imported into Cytoscape 3.9 software to construct the herb-component-target network.

### 2.4. Dyslipidemia PPI Network Construction

The targets of dyslipidemia treatment were entered into the BisoGenet plug-in in Cytoscape 3.7.1 software to identify the dyslipidemia protein-protein interaction (PPI) network, with the organism set to *Homo sapiens* and the biorelation type set to protein-protein interaction. The network was later analysed by the CytoNCA plug-in to screen out the core dyslipidemia PPI network.

### 2.5. Construction of the HLJDD-Dyslipidemia PPI Network

The targets of HLJDD and dyslipidemia treatment were imported into jvenn (http://jvenn.toulouse.inra.fr/app/example.html, 2021/09/20). A Venn diagram with the common targets of HLJDD and dyslipidemia treatment was obtained.

The common targets were then imported into the STRING database (https://www.string-db.org/, 2021/09/25) to obtain the HLJDD-dyslipidemia PPI network, with the organism set to *Homo sapiens*, and the minimum required interaction score was set to medium confidence (0.400). Text mining, experiments, and databases were selected as the interaction sources.

The network was imported into Cytoscape 3.9 software to screen out the core HLJDD-dyslipidemia PPI network through the maximal clique centrality (MCC) algorithm in the CytoHubba plug-in.

### 2.6. Enrichment Analysis

The *R* package “ClusterProfiler” (http://www.bioconductor.org/, 2021/12/10) was used to carry out gene ontology (GO) enrichment analysis and Kyoto Encyclopedia of Genes and Genomes (KEGG) pathway enrichment analysis of common targets of HLJDD and dyslipidemia treatment. The GO enrichment analysis items were the biological process (BP), cellular component (CC), and molecular function (MF). The organism was set to *Homo sapiens*, and the *P* value was set to ≤0.05.

The article "Study on the Mechanism of Huanglian Jiedu Decoction in Treating Dyslipidemia Based on Network Pharmacology" was published in 2022. Journal: J Healthc Eng.

### 2.7. Herb-Component-Target-KEGG Pathway Network Construction

The affiliation between herbs, components, common targets, and the top 30 enriched KEGG pathways were further imported to Cytoscape 3.9 software to construct the herb-component-target-KEGG pathway network. The network was analysed using the network analysis function.

## 3. Results

### 3.1. Herb-Component-Target Network Analysis

Four herbs, 22 components, and 234 targets of HLJDD were retrieved from TCMSP. The herb-component-target network (Figure 2) showed the relationship between herbs, components, and targets. HLJDD may exert its effects through these targets.

### 3.2. Dyslipidemia PPI Network Analysis

A total of 221 targets of dyslipidemia treatment were retrieved from the GeneCards, OMIM, PharmGKB, TTD, and DrugBank databases. The dyslipidemia PPI network (Figure 3(a)) showed the interaction between targets related to dyslipidemia treatment, with 4381 nodes and 104818 edges. The CytoNCA plug-in in Cytoscape 3.7.1 software was used to analyse the network and screen out nodes with a degree centrality (DC) larger than twice the median (Figure 3(b)). On this basis, the top 10% of nodes with the highest betweenness centrality (BC), closeness centrality (CC), and DC were screened out to obtain the core dyslipidemia PPI network (Figure 3(c)).

### 3.3. HLJDD-Dyslipidemia PPI Network Analysis

Thirty-one common targets of HLJDD and dyslipidemia treatment were obtained and are shown in a Venn diagram (Figure 4(a)). The HLJDD-dyslipidemia PPI network (Figure 4(b)) shows the interactions among the common targets. The core network of the HLJDD-dyslipidemia PPI network (Figure 4(c)) shows the top 10 core targets of the HLJDD-dyslipidemia PPI network: IL-6, TNF, NOS3, PTGS2, SERPINE1, VCAM1, CXCL8, HMOX1, IL-10, and ACE. These may be the potential key targets of HLJDD for dyslipidemia treatment.

### 3.4. Enrichment Analysis

GO enrichment and KEGG pathway enrichment analyses of the common targets of HLJDD and dyslipidemia treatment were performed using the *R* package “ClusterProfiler.”

Bioinformatics annotation of these genes identified 1058 GO terms. The analysis results of the GO functions including the top 10 enriched biological processes, CCs, and MFs are shown in a bubble chart (Figures 5(a)–5(c)). Regarding the biological processes, the common targets were mainly enriched in the regulation of DNA-binding transcription factor activity, regulation of lipid localization, positive regulation of DNA-binding transcription factor activity, reactive oxygen species metabolic process, regulation of inflammatory response, positive regulation of the small-molecule metabolic process, regulation of blood pressure, negative regulation of lipid localization, lipid storage, and negative regulation of lipid storage. For cellular components, the targets were enriched in the external side of the plasma membrane, membrane raft, membrane microdomain, caveola, plasma membrane raft, endoplasmic reticulum lumen, secretory granule lumen, cytoplasmic vesicle lumen, vesicle lumen, and transcription preinitiation complex. For molecular function, the targets were enriched in nuclear receptor activity, ligand-activated transcription factor activity, DNA-binding transcription factor binding, transcription coactivator binding, transcription coregulator binding, steroid binding, haem binding, tetrapyrrole binding, steroid hormone receptor activity, and RNA polymerase II general transcription initiation factor binding.

The article "Study on the Mechanism of Huanglian Jiedu Decoction in Treating Dyslipidemia Based on Network Pharmacology" was published in 2022. Journal: J Healthc Eng.

The KEGG pathway analysis revealed the presence of 64 enriched KEGG pathways, which are shown in a bubble chart (Figure 5(d)). The pathways include the AGE-RAGE signalling pathway in diabetic complications, fluid shear stress and atherosclerosis, chemical carcinogenesis-receptor activation, Chagas disease, insulin resistance, nonalcoholic fatty liver disease, lipids and atherosclerosis, malaria, viral protein interaction with cytokines and cytokine receptors, the NF-kappa B signalling pathway, the HIF-1 signalling pathway, diabetic cardiomyopathy, human cytomegalovirus infection, African trypanosomiasis, pertussis, hypertrophic cardiomyopathy, rheumatoid arthritis, the IL-17 signalling pathway, amoebiasis, the C-type lectin receptor signalling pathway, the TNF signalling pathway, the FoxO signalling pathway, *Yersinia* infection, alcoholic liver disease, the intestinal immune network for IgA production, legionellosis, inflammatory bowel disease, chemical carcinogenesis-DNA adducts, the PPAR signalling pathway, and leishmaniasis.

These GO functions and pathways may be the potential mechanisms of HLJDD in dyslipidemia treatment.

### 3.5. Herb-Component-Target-KEGG Pathway Network Analysis

The relationships between herbs, components, common targets of HLJDD and dyslipidemia treatment, and enriched KEGG pathways are shown in Figure 6. The network contains 4 herbs, 14 components, 31 common targets between HLJDD and dyslipidemia treatment, and the top 30 enriched KEGG pathways. According to the data generated in this study, the herbs with the highest DC were Radix Scutellariae and Cortex Phellodendri. Quercetin, kaempferol, berberine, acetic acid, and wogonin were predicted to be the major compounds in HLJDD related to dyslipidemia. Among the potential targets, TNF, IL-6, IL-8, PTGS2, and IL-10 had relatively more connected edges. Among the pathways, the AGE-RAGE, NF-*κ*B, HIF-1, IL-17, TNF, FoxO, and PPAR signalling pathways are closely related to the treatment of dyslipidemia with HLJDD.

The article "Study on the Mechanism of Huanglian Jiedu Decoction in Treating Dyslipidemia Based on Network Pharmacology" was published in 2022. Journal: J Healthc Eng.

## 4. Discussion

Dyslipidemia is a major risk factor for atherosclerotic CVD, which has become the leading cause of death worldwide. TCM recipes exert therapeutic effects on several incurable diseases, including dyslipidemia [12]. However, many studies still apply the conventional research approach of “one drug, one target, and one illness,” which does not account for the multitarget and multicomponent characteristics of TCM recipes. Due to the development of bioinformatics, the network approach has become a novel means of efficiently and systemically identifying the potential molecular mechanisms of TCM recipes [14].

In the present study, several network-based computational methods and algorithm-based approaches were used to predict targets and construct networks to assess the molecular interactions associated with HLJDD when used as a dyslipidemia therapy. Our research showed that some of the compounds in HLJDD such as quercetin, berberine, and kaempferol played a dyslipidemia-regulating role. We also showed that the biological functions of HLJDD-regulating dyslipidemia were related to DNA-binding transcription factor activity, lipid localization and storage, reactive oxygen species metabolic process, and inflammatory response.

Many genes such as APOB, LPL, APOA1, LEP, CD36, IL-6, and APOE may play an important role in dyslipidemia. Analysis of the functions of these genes may expand our understanding of the fundamental mechanisms leading to dyslipidemia. Apolipoprotein B (APOB) is associated with dyslipidemia and atherosclerosis development [15]. Even in the absence of other risk factors, elevated levels of lipoproteins containing APOB can drive the development of atherosclerosis in humans and animals [16]. These APOB-containing lipoproteins also bind exchangeable apolipoproteins such as APOA1 and APOE, which are regulated by lipoprotein lipase (LPL) and CD36 and are involved in the process [17, 18]. Moderate dyslipidemia and dyslipoproteinemia have been reported to elevate inflammatory markers such as TNF-*α* and IL-6 concentrations, and inflammation slowly induces an increase in myeloperoxidase concentration, which decreases APOAI and HDL-C levels and disturbs HDL function, which confirms that inflammation plays an important role in dyslipidemia [19]. LEP is a protein hormone that has been widely shown to participate in the regulation of sugar, fat, and energy metabolism [20, 21]. In summary, the interaction of disease networks plays a key role in dyslipidemia.

The article "Study on the Mechanism of Huanglian Jiedu Decoction in Treating Dyslipidemia Based on Network Pharmacology" was published in 2022. Journal: J Healthc Eng.

It has been reported that many compounds of HLJDD regulate dyslipidemia. The analysis of the network revealed that quercetin, kaempferol, berberine, acetic acid, and wogonin are predicted to be the major compounds in HLJDD for treating dyslipidemia. Several studies have shown that quercetin, an effective antioxidant and free radical scavenger against oxidative stress, has a hypolipidemic effect and antioxidative role by inhibiting ROS overgeneration and lipid peroxidation in mitochondria [22–24]. In addition, quercetin suppresses inflammatory enzymes including cyclooxygenase and lipoxygenase, as well as proinflammatory mediators [25]. To date, only a proprietary formulation of three naturally occurring substances with putative complementary lipid-lowering properties exists, one of which is berberine combined with folic acid, which has been extensively investigated in several randomized controlled trials [26]. A large body of literature supports different pharmacological actions of berberine such as antidiabetic, antiobesity, hypotensive, and hypolipidemic properties, which could be interesting in the management of patients with a high CVD risk [27]. Kaempferol showed slight inhibition of cholesterol and effectively prevented atherosclerosis induced by high cholesterol [28, 29]. Studies have also confirmed that wogonin may have beneficial effects in ameliorating dyslipidemia via PPAR*α* activation. Furthermore, other compounds of HLJDD also have the function of regulating dyslipidemia, such as crocetin [30], baicalein [31], and geniposide [32]. Together, they form a network that embodies the multicompound role of the TCM decoction in regulating dyslipidemia.

The analysis of the network showed that the biological functions of HLJDD were linked to DNA-binding transcription factor activity, lipid localization and storage, reactive oxygen species metabolic process, and inflammatory response, which are closely related to the pathological mechanism of lipid metabolism. The results of KEGG analysis indicated that the AGE-RAGE, NF-*κ*B, HIF-1, IL-17, TNF, FoxO, and PPAR signalling pathways were enriched in the antidyslipidemic action of HLJDD. It has been reported that the AGE-RAGE-oxidative stress axis is involved in the onset and progression of metabolic syndrome induced by a high-fructose diet [33]. Quercetin may have a role in the management of metabolic disorders via different mechanisms, such as increasing adiponectin and decreasing leptin and antioxidant activity through the NF-*κ*B signalling pathway [23]. Animal experiments have shown that the main active ingredient of HLJDD, berberine, can regulate metabolic homeostasis and suppress adipose tissue fibrosis by inhibiting the expression of the HIF-1 signalling pathway [34]. This result demonstrates the multipathway characteristics of herbal formulas in the treatment of diseases.

The article "Study on the Mechanism of Huanglian Jiedu Decoction in Treating Dyslipidemia Based on Network Pharmacology" was published in 2022. Journal: J Healthc Eng.

In this study, we found that the active ingredients of HLJDD including quercetin, kaempferol, berberine, acetic acid, and wogonin may act on multiple targets such as TNF, IL-6, IL-8, PTGS2, and IL-10 and regulate multiple signalling pathways such as the AGE-RAGE, NF-*κ*B, HIF-1, IL-17, and PPAR signalling pathways to regulate lipid localization and storage, reactive oxygen species metabolic processes, and inflammatory responses, thereby achieving the treatment of dyslipidemia.

This study employed the method of network pharmacology and clearly revealed the “multicomponent, multitarget, and multipathway” mechanism of HLJDD in treating dyslipidemia through network construction. In the future, clinical trials and animal experiments will be conducted based on previous reports [35, 36] to further analyse and validate the mechanism of HLJDD in combating dyslipidemia identified in this study.

## Figures and Tables

**Figure 1:** Illustration of the study strategy.

**Figure 2:** Herb-component-target network.

**Figure 3:** Dyslipidemia PPI network. (a) Nodes with a DC larger than twice the median are highlighted in red. (b) The top 10% of nodes with the highest BC, CC, and DC are highlighted in yellow. (c) Core dyslipidemia PPI network.

**Figure 4:** (a) Venn diagram of HLJDD and dyslipidemia treatment. (b) HLJDD-dyslipidemia PPI network. (c) Core HLJDD-dyslipidemia PPI network.

**Figure 5:** Enrichment analysis. (a) Biological process (BP), (b) cellular component (CC), and (c) molecular function (MF) of GO enrichment analysis. (d) KEGG pathway enrichment analysis.

**Figure 6:** Herb-component-target-KEGG pathway network of herbs and components, common targets of HLJDD and dyslipidemia treatment, and the top 30 enriched KEGG pathways.

## Data Availability

The data used to support the findings of this study are available from the corresponding authors upon request.

## References

[1] Duggan J. P., Peters A. S., Trachiotis G. D., Antevil J. L. (2022). Epidemiology of coronary artery disease. *Surgical Clinics of North America*.

[2] Du H., Shi Q., Song P. (2022). Global burden attributable to high low-density lipoprotein-cholesterol from 1990 to 2019. *Frontiers in cardiovascular medicine*.

[3] Li J. J., Liu H. H., Li S. (2022). Landscape of cardiometabolic risk factors in Chinese population: a narrative review. *Cardiovascular Diabetology*.

The article "Study on the Mechanism of Huanglian Jiedu Decoction in Treating Dyslipidemia Based on Network Pharmacology" was published in 2022. Journal: J Healthc Eng.

[4] Yeung E., Daniels S. R., Patel S. S. (2021). Dyslipidemia in childhood and adolescence: from screening to management. *Current Opinion in Endocrinology Diabetes and Obesity*.

[5] Ferraro R. A., Leucker T., Martin S. S., Banach M., Jones S. R., Toth P. P. (2022). Contemporary management of dyslipidemia. *Drugs*.

[6] Ma Y. L., Yao H., Yang W. J., Ren X. X., Teng L., Yang M. C. (2017). Correlation between traditional chinese medicine constitution and dyslipidemia: a systematic review and meta-analysis. evidence-based complementary and alternative medicine. *eCAM*.

[7] Rauf A., Akram M., Anwar H. (2022). Therapeutic potential of herbal medicine for the management of hyperlipidemia: latest updates. *Environmental Science and Pollution Research*.

[8] Lee Y. S., Lee J. M., Chung H., Woo J. S., Lee B. C., Kim W. (2022). Efficacy and safety of da-chai-hu-tang in lipid profiles in high-risk, statin-treated patients with residual HyperTG: a 12-week, randomized, active-control, open clinical study. *The Life*.

[9] Chen J., Ye C., Yang Z. (2022). Effects of erchen decoction on oxidative stress-related cytochrome P450 metabolites of arachidonic acid in dyslipidemic mice with phlegm-dampness retention syndrome: a randomized, controlled trial on the correspondence between prescription and syndrome. *Evidence-based Complementary and Alternative Medicine*.

[10] Xu Z., Sheng Y., Zeng G. (2021). Metabonomic study on the plasma of high-fat diet-induced dyslipidemia rats treated with Ge gen qin lian decoction by uplcms. *Evidence-based Complementary and Alternative Medicine*.

[11] Feng W., Ye X., Lv H., Hou C., Chen Y. (2019). Wendan decoction for dyslipidemia: protocol for a systematic review and meta-analysis. *Medicine*.

[12] Effectiveness and safety of Hwangryunhaedok-Tang (Huang-Lian-Jie-Du-Tang (2021). Oren-Gedoku-to) for dyslipidemia: a protocol for a PRISMA-compliant systematic review and meta-analysis: Erratum. *Medicine*.

[13] Cai Y., Wen J., Ma S. (2021). Huang-lian-jie-du decoction attenuates atherosclerosis and increases plaque stability in high-fat diet-induced ApoE(-/-) mice by inhibiting M1 macrophage polarization and promoting M2 macrophage polarization. *Frontiers in Physiology*.

[14] Cui Y., Wang H., Wang D. (2021). Network pharmacology analysis on the mechanism of huangqi sijunzi decoction in treating cancer-related fatigue. *Journal of healthcare engineering*.

[15] Sniderman A., Langlois M., Cobbaert C. (2021). Update on apolipoprotein B. *Current Opinion in Lipidology*.

[16] Sniderman A. D., Thanassoulis G., Glavinovic T. (2019). Apolipoprotein B particles and cardiovascular disease: a narrative review. *JAMA cardiology*.

The article "Study on the Mechanism of Huanglian Jiedu Decoction in Treating Dyslipidemia Based on Network Pharmacology" was published in 2022. Journal: J Healthc Eng.

[17] Whitacre B. E., Howles P., Street S., Morris J., Swertfeger D., Davidson W. S. (2022). Apolipoprotein E content of VLDL limits LPL-mediated triglyceride hydrolysis. *Journal of Lipid Research*.

[18] Zeng Z., Cao B., Guo X. (2018). Apolipoprotein B-100 peptide 210 antibody inhibits atherosclerosis by regulation of macrophages that phagocytize oxidized lipid. *American Journal of Tourism Research*.

[19] Kimak E., Zięba B., Duma D., Solski J. (2018). Myeloperoxidase level and inflammatory markers and lipid and lipoprotein parameters in stable coronary artery disease. *Lipids in Health and Disease*.

[20] Socol C. T., Chira A., Martinez-Sanchez M. A. (2022). Leptin signaling in obesity and colorectal cancer. *International Journal of Molecular Sciences*.

[21] Tam B. T., Murphy J., Khor N., Morais J. A., Santosa S. (2020). Acetyl-CoA regulation, OXPHOS integrity and leptin levels are different in females with childhood vs adulthood onset of obesity. *Endocrinology*.

[22] Derakhshanian H., Djalali M., Djazayery A. (2020). Quercetina Melhora o Perfil Lipídico e Apolipoproteico em Ratos Tratados com Glicocorticóides em Altas Doses. *Arquivos Brasileiros de Cardiologia*.

[23] Hosseini A., Razavi B. M., Banach M., Hosseinzadeh H. (2021). Quercetin and metabolic syndrome: a review. *Phytotherapy Research*.

[24] Villarroel-Vicente C., Gutiérrez-Palomo S., Ferri J., Cortes D., Cabedo N. (2021). Natural products and analogs as preventive agents for metabolic syndrome via peroxisome proliferator-activated receptors: an overview. *European Journal of Medicinal Chemistry*.

[25] Mirsafaei L., Reiner Ž, Shafabakhsh R., Asemi Z. (2020). Molecular and biological functions of quercetin as a natural solution for cardiovascular disease prevention and treatment. *Plant Foods for Human Nutrition*.

[26] Barrios V., Escobar C., Cicero A. F. G. (2017). A nutraceutical approach (Armolipid Plus) to reduce total and LDL cholesterol in individuals with mild to moderate dyslipidemia: review of the clinical evidence. *Atherosclerosis Supplements*.

[27] Tabeshpour J., Imenshahidi M., Hosseinzadeh H. (2017). A review of the effects of Berberis vulgaris and its major component, berberine, in metabolic syndrome. *Iranian journal of basic medical sciences*.

[28] Feng Z., Wang C., Yue (2021). Kaempferol-induced GPER upregulation attenuates atherosclerosis via the PI3K/AKT/Nrf2 pathway. *Pharmaceutical Biology*.

[29] Ochiai A., Othman M. B., Sakamoto K. (2021). Kaempferol ameliorates symptoms of metabolic syndrome by improving blood lipid profile and glucose tolerance. *Bioscience Biotechnology & Biochemistry*.

The article "Study on the Mechanism of Huanglian Jiedu Decoction in Treating Dyslipidemia Based on Network Pharmacology" was published in 2022. Journal: J Healthc Eng.

[30] Diao S. L., Sun J. W., Ma B. X., Li X. M., Wang D. (2018). Influence of crocetin on high-cholesterol diet induced atherosclerosis in rats via anti-oxidant activity together with inhibition of inflammatory response and p38 MAPK signaling pathway. *Saudi Journal of Biological Sciences*.

[31] Baradaran Rahimi V., Askari V. R., Hosseinzadeh H. (2021). Promising influences of Scutellaria baicalensis and its two active constituents, baicalin, and baicalein, against metabolic syndrome: a review. *Phytotherapy Research*.

[32] Zheng Y., Xiao Y., Zhang D. (2021). Geniposide ameliorated dexamethasone-induced cholesterol accumulation in osteoblasts by mediating the GLP-1R/ABCA1 Axis. *Cells*.

[33] Cannizzaro L., Rossoni G., Savi F. (2017). Regulatory landscape of AGE-RAGE-oxidative stress axis and its modulation by PPAR*γ* activation in high fructose diet-induced metabolic syndrome. *Nutrition & Metabolism*.

[34] Hu M., Wu F., Luo J. (2018). The role of berberine in the prevention of HIF-1*α* activation to alleviate adipose tissue fibrosis in high-fat-diet-induced obese mice. *Evidence-based Complementary and Alternative Medicine*.

[35] Upadya H., Prabhu S., Prasad A., Subramanian D., Gupta S., Goel A. (2019). A randomized, double blind, placebo controlled, multicenter clinical trial to assess the efficacy and safety of Emblica officinalis extract in patients with dyslipidemia. *BMC Complementary and Alternative Medicine*.

[36] Peng C. H., Yang M. Y., Yang Y. S., Yu C. C., Wang C. J. (2017). Antrodia cinnamomea prevents obesity, dyslipidemia, and the derived fatty liver via regulating AMPK and SREBP signaling. *The American Journal of Chinese Medicine*.

